# Multimodality Imaging *In Vivo* for Preclinical Assessment of Tumor-Targeted Doxorubicin Nanoparticles

**DOI:** 10.1371/journal.pone.0034463

**Published:** 2012-04-03

**Authors:** Jae Youn Hwang, Jinhyoung Park, Bong Jin Kang, David J. Lubow, David Chu, Daniel L. Farkas, K. Kirk Shung, Lali K. Medina-Kauwe

**Affiliations:** 1 Department of Biomedical Sciences, Cedars-Sinai Medical Center, Los Angeles, California, United States of America; 2 Department of Biomedical Engineering, University of Southern California, Los Angeles, California, United States of America; 3 Department of Medicine, University of California Los Angeles Geffen School of Medicine, Los Angeles, California, United States of America; Case Western Reserve University, United States of America

## Abstract

This study presents a new multimodal imaging approach that includes high-frequency ultrasound, fluorescence intensity, confocal, and spectral imaging to improve the preclinical evaluation of new therapeutics *in vivo*. Here we use this approach to assess *in vivo* the therapeutic efficacy of the novel chemotherapy construct, HerDox during and after treatment. HerDox is comprised of doxorubicin non-covalently assembled in a viral-like particle targeted to HER2+ tumor cells, causing tumor cell death at over 10-fold lower dose compared to the untargeted drug, while sparing the heart. Whereas our initial proof-of-principle studies on HerDox used tumor growth/shrinkage rates as a measure of therapeutic efficacy, here we show that multimodal imaging deployed during and after treatment can supplement traditional modes of tumor monitoring to further characterize the particle in tissues of treated mice. Specifically, we show here that tumor cell apoptosis elicited by HerDox can be monitored *in vivo* during treatment using high frequency ultrasound imaging, while *in situ* confocal imaging of excised tumors shows that HerDox indeed penetrated tumor tissue and can be detected at the subcellular level, including in the nucleus, via Dox fluorescence. In addition, ratiometric spectral imaging of the same tumor tissue enables quantitative discrimination of HerDox fluorescence from autofluorescence *in situ*. In contrast to standard approaches of preclinical assessment, this new method provides multiple/complementary information that may shorten the time required for initial evaluation of *in vivo* efficacy, thus potentially reducing the time and cost for translating new drug molecules into the clinic.

## Introduction

Different types of radiation, including light, radio-waves, ultrasound, x-rays, and gamma rays, have all been utilized to image the structure and function of tissues of interest inside a living object. Each imaging modality offers different spatial and temporal resolutions as well as different sensitivities in measurement of morphological or functional properties of tissues [1], [2]. Therefore, the simultaneous use of different imaging modalities should combine the strengths while reducing the shortcomings inherent to each individual modality, thus allowing enhanced diagnosis, therapeutic monitoring, and improved preclinical research. Because of the aforementioned advantages, noninvasive multimodal imaging based on optical, ultrasound, magnetic resonance imaging (MRI), computerized-tomography (CT), single-photon emission computed tomography (SPECT), and positron emission tomography (PET) is now not only becoming standard practice in the clinic, but also a rapidly emerging technique for a variety of *in vivo* preclinical studies, from molecular pharmacology to stem cell research [1], [3]–[12].

To date, much effort has been focused on the development of non-invasive multimodal imaging approaches, aimed at visualizing diseased lesions and monitoring stem cell migration. For instance, tumor angiogenesis has been detected and monitored using intravital confocal, MRI, and optical imaging simultaneously with novel multimodal quantum dots [10], whereas breast cancer micro-calcifications have been detected using dual modality SPECT/NIR fluorescence imaging [13]. In addition, PET and bioluminescence imaging have been simultaneously employed to noninvasively monitor implanted neural progenitor cells and their migrations [7], [14]. Moreover, multimodal imaging can enable improved identification of new drug candidates by detecting enhanced efficiency, thus reducing cost and time for drug development [15], [16].

We have previously developed the viral capsid-derived fusion protein, HerPBK10, which targets noncovalently attached therapeutic molecules to human epidermal growth factor receptor 2- positive (HER2+) cells, including breast, ovarian, and glioma cancer cells, and mediates penetration into the tumor cells, resulting in tumor-targeted toxicity [17]–[23]. Our recent studies have shown that the tumor-targeted gallium corrole, HerGa (which results from the spontaneous, non-covalent assembly of the sulfonated gallium corrole, S2Ga, and HerPBK10), exhibits intense fluorescence and cytotoxicity to HER2+ MDA-MB-435 cancer cells, thus enabling both tumor detection and elimination [17]–[19]. In those studies, we for the first time employed a multimode optical imaging system, specifically using fluorescence intensity, spectral, lifetime, and two-photon excited fluorescence imaging modes, to assess HerGa *in vivo*. This multimode optical imaging *in vivo* allowed us to monitor the kinetics of the drug molecule accumulation in small animals as well as specifically and quantitatively characterize the *in vivo* micro-environment surrounding the drug with micro- to macro-scopic resolution [24], [25]. More recently, we have developed another novel chemotherapy particle, HerDox, which is a non-covalent assembly of doxorubicin with HerPBK10. That study showed that HerDox allows doxorubicin potency to remain unaltered during assembly, transport, and release into target cells while enabling lower drug dose for tumor killing, thus improving the safety of doxorubicin over standard untargeted treatment that is used in the clinic [26]. As the carrier protein used in both HerGa and HerDox can be modified to target other tumor types, we have recently explored the possibility of whether preclinical evaluation of such targeted particles can be expedited through new combination of multiple imaging modalities.

In the present study, we for the first time combined four imaging modalities (Fig. 1), including high-frequency ultrasound, fluorescence intensity, confocal, and ratiometric spectral imaging [25], in order to characterize our tumor-targeted doxorubicin nanoparticles *in vivo* and *ex vivo*. High-frequency ultrasound imaging provides tissue microanatomy with better spatial resolution than standard ultrasound imaging, thus enabling one to monitor structural changes of the regions of interest, including cell apoptosis *in vivo*. In contrast, fluorescence intensity imaging is suited for continuous tracking of movements and concentrations of labeled molecules *in vivo* and *ex vivo*, based on the spatial distribution of intensity, thus monitoring the effects of drug candidates on the target pathology. Ratiometric spectral imaging provides quantitative spectral signatures at every pixel of an image, allowing one to discriminate between the background (autofluorescence) and fluorescence of interest more quantitatively and specifically [26]. Confocal microscopy provides better depth-selectivity imaging than standard fluorescence microscopy, thus identifying the localization of molecules in tissues with high resolution [24]. The combination of these imaging modes compared to using a single imaging mode alone offers multiple/complementary information, thus enabling better *in vivo* characterization of nanoparticles such as the ones tested here. In this study, tumor response to HerDox treatment was quantitatively monitored *in vivo* using high-frequency ultrasound imaging, and cell death was verified using confocal fluorescence imaging of immunostained tumor sections extracted from HerDox-treated and untreated mice. In addition, we verified the tumor-preferential biodistribution of HerDox using fluorescence intensity imaging, and analyzed specific accumulation and localization in tumors *in situ* using high-resolution confocal and spectral imaging and analysis. These results demonstrate that the multimodal imaging approach presented here is suited for the assessment of new chemotherapy nanoparticles as a novel alternative to standard, single-mode imaging.

**Figure 1:** Multimodality imaging for preclinical assessment of nanoparticles and information provided by each modality.

## Materials and Methods

### Ethics Statement

All *in vivo* and euthanasia procedures in this study were carried out in strict accordance with the recommendations in the Guide for the Care and Use of Laboratory Animals of the National Institutes of Health. The protocol was approved by the Cedars-Sinai Medical Center Institutional Animal Care and Use Committee (IACUC) (Protocol Number: 2794). All efforts were made to minimize suffering.

### Materials

The MDA-MB-435 human HER2+ tumor cell line was obtained from the National Cancer Institute, and maintained in DMEM, 10% fetal bovine serum under 5% CO2. Doxorubicin-HCI was purchased from Sigma-Aldrich. HBS, HEPES-buffered saline (20 mM HEPES, pH 7.5; 150 mM NaCl); PBS, phosphate-buffered saline. For TUNEL staining of tumor sections, an *in situ* cell death detection kit was purchased from Roche Applied Science (IN, USA).

### Animals

Female immunodeficient (nu/nu) mice (6–8 weeks; Charles River Laboratories International, Wilmington, MA, USA) received subcutaneous bilateral flank injections of 1×10^7^ MDA-MB-435 cells/injection to create a xenograft tumor model, and tumor growth monitored by measuring tumor volume via calipers. Treatments were initiated after tumors reached ∼200–300 mm^3^.

### HerDox assembly

The viral capsid-derived fusion protein, HerPBK10, was assembled with doxorubicin following established procedures [26]. Briefly, complementary oligonucleotide duplexes were incubated with Dox at 1∶10 molar ratio of DNA∶Dox at room temperature (RT) for 30 minutes, followed by incubation with HerPBK10 at 6∶1 molar ratio of HerPBK10∶DNA-Dox in HBS, followed by ultrafiltration using 50 k MW cutoff (mwco) filter membranes to isolate HerDox from incompletely assembled components. The Dox concentration in HerDox was determined by extrapolating the measured absorbance at 480 nm or fluorescence at 590 nm (Ex: 480 nm) against a Dox absorbance or fluorescence calibration curve (SpctraMax, Molecular Devices, USA). HerDox dose is based on the concentration of Dox in HerDox.

### HerDox and Dox tail-vein administration

∼200 µl of HerDox at 1 µM (0.004 mg/kg) and ∼200 µl of HerDox at 10 µM (0.04 mg/kg), in which the injection volume was dependent on the weight of mice (28–30 g), were injected daily into mice (HerDox: n = 3, Dox: n = 3, and untreated: n = 3) through the tail-vein using 3/10cc insulin syringe (Needle size: 29_G_ ½″) for six sequential days. Mice were anesthetized before tail-vein injections following IACUC-approved procedures.

### High-frequency ultrasound imaging

A custom-built ultrasound bio-microscope (UBM) was utilized for high-frequency ultrasound imaging. A 40 megahertz (MHz) LiNbO_3_ light-weight single-element ultrasound transducer, with a fixed focal distance at 6 mm and bandwidth of 75%, was used to scan the tumor regions of treated mice [27]. The transmission signal emitted from the transducer was a three cycle sine burst of 50 MHz with 80 V peak-to-peak voltage. Importantly, the transmission condition was maintained during the evaluation of HerDox efficacy for the tumor treatment.

Ultrasound images of tumor regions *in vivo* were obtained before drug (HerDox and Dox) administration, after the third daily intravenous (IV) administration, and 24 h after the last (sixth) daily IV administration to the tumor-bearing mice (three mice, or six tumors, per group) respectively. Here, the dose of Dox at 0.04 mg/kg/day was chosen as a positive control since this dose of untargeted Dox exhibits similar efficacy on tumor treatment to the dose of HerDox at 0.004 mg/kg/day [26]. The transducer covered by a Tegaderm™ transparent dressing (3 M, St. Paul, MN) was coupled to the skin after an ultrasonic gel was generously spread on the surface of the transducer for the *in vivo* imaging. After ultrasound signals were transmitted to the tumor sites, ultrasound echo signals from the sites were detected by the transducer and post-processed using a program we developed (Matlab R2010b, Mathworks) to construct ultrasound images. During each measurement at the indicated time points, an almost identical tumor site of each mouse was placed at the focal distance of the transducer. In addition, the tumors were harvested from the mice, and then imaged in order to examine the echo intensity changes in the *ex vivo* tumors (4 tumors per group) after the drug treatment.

For the quantitative analysis, we calculated the mean intensities of ultrasound echo signal from tumor regions in the images obtained at indicated time-points *in vivo* and *ex vivo* and compared the mean intensities of tumors before and after the HerDox and Dox treatment.

### Fluorescence intensity imaging *ex vivo*

Fluorescence intensity imaging of tumors and specific organs (including the liver, kidney, spleen, heart, and skeletal muscle) was performed by harvesting tissues from euthanized mice 24 h after the mice received daily tail vein injections of 0.004 mg/kg HerDox for 6 consecutive days. A multimode optical imaging system that we previously developed [24] was used here for the fluorescence intensity imaging *ex vivo*. For excitation of HerDox, 532 nm laser light (CrystaLaser, up to ∼0.5 W), which provides better tissue penetration than 488 nm laser light [28], was delivered onto specimens through several mirrors and diffusers, and then emission light from the specimens was filtered through an emission filter (590±30 nm), and recorded in a high-sensitivity cooled CCD camera (PIXIS 400, Princeton Instruments, quantum efficiency at 590 nm: ∼95%). After the fluorescence images were acquired, background subtraction of the images was performed using ImageJ to reduce artifacts resulting from the laser beam profile. It is noted that although the light wavelength utilized here was not perfectly matched with the typical maximum absorption wavelengths (∼480–490 nm) for excitation of Dox, light at 532 nm is still capable of considerable (fraction with respect to the maximum absorbance: 0.86) Dox excitation in tissues [26].

### *In situ* confocal/spectral imaging and analysis

The *in situ* confocal imaging was performed using a Leica SPE confocal microscope with a 488 nm laser light delivered onto the tumors for excitation of HerDox, while the fluorescence from the tumors was collected by a 40× ACS oil objective. Fluorescence within 550–600 nm was selected by an acousto-optic tunable filter (AOTF) and recorded in a photomultiplier tube incorporated in the microscope. A total of 18 confocal fluorescence images of HerDox-treated, Dox-treated, and untreated tumors were acquired at sequential z-depths within 36 µm with a step size of 2 µm respectively. A maximum intensity z-projection of the images was performed, and then mean fluorescence intensities of the images were measured using ImageJ software.

### Ratiometric spectral imaging and analysis with spectral unmixing

For ratiometric spectral imaging and analysis, which offers a more quantitative analysis than standard spectral imaging in chemotherapy assessment [25], 15 images of the HerDox-treated and untreated tumors at a specified depth were acquired within the spectral range of 510–650 nm, with a step size of 10 nm, while HerDox was excited by 488 nm light using a Leica SPE confocal microscope. Reference spectral signatures were created through combination of different ratios of a pure doxorubicin and auto-fluorescence spectral signature. Here it is important to note that there is no significant difference between the spectral signatures of HerDox and Dox fluorescence to have any significant effects on separating doxorubicin from autofluorescence [26]. Therefore, we utilized the spectral signature of free doxorubicin to perform the ratiometric spectral imaging and analysis. While the pure spectral signature of doxorubicin was acquired from an image cube (spectral range: 510–650 nm, a step size: 10 nm), obtained by spectral imaging of 100 µM doxorubicin solution using the Leica SPE confocal microscope, the autofluorescence spectral signature was acquired from an image cube (spectral range: 510–650 nm, a step size: 10 nm) obtained by spectral imaging of untreated tumors [25]. Here four reference spectral signatures (pure autofluorescence, 0.1·doxorubin+0.9·autofluorescence, 0.2· doxorubicin+0.8·autofluorescence, 0.3·doxorubin+0.7·autofluorescence) were generated for the classification using a program we previously developed [25], as the reference spectral signatures with higher ratio of doxorubicin more than 0.4 relative to autofluorescence did not have any significant effects on spectral classification (equation for generating the mixed spectral signatures: *S* = *a*_1_×*A*+*a*_2_×*H*, where *S* is the composite spectral signature, *A* and *H* are the spectral signatures of autofluorescence and Dox fluorescence respectively, and *a_n_* is the relative contribution of the signals). The spectral classification of the images as defined by the reference spectral signatures was performed based on Euclidean distance measure using a program we previously developed [25]. Furthermore, linear spectral unmixing of those images was performed by using a spectral unmixing program (plug-in in ImageJ we developed), for comparison to the ratiometric spectral imaging and analysis.

### H&E and TUNEL imaging

For TUNEL staining of the sections of tumors extracted from the mice treated with different drug molecules, the unstained sections were dewaxed and hydrated by the following procedures; 1) sections were incubated in dry oven 60 deg for 1 hour; 2) submerged in xylenes for 4 min, 5 times; 3) hydrated by submerging in 100%, 95%, 90%, 80%, 70% ethanol for 3 min, 2 times each; 4) submerged in 100% water. After the dewax and hydration of the sections, epitope retrieval of the sections was performed with Proteinase K (20 ug/ml in 10 mM Tris pH 7.8), and then followed by TUNEL staining using the *in situ* cell death detection kit (following the manufacturer's procedures; Roche applied science, Indianapolis, IN, USA) after the sections were rinsed with PBS. After TUNEL staining of the tumor sections, confocal fluorescence imaging of the sections was performed using a Leica confocal SPE microscope (20×, ex: 488 nm, and em: 530 nm). In addition, the hematoxilin and eosin (H&E) sections, prepared by the Pathology Service at the Cedars-Sinai Medical Center, were imaged using an Olympus microscope (IX71) incorporating a CCD camera (QImaging, RETIGA EXI) and a liquid crystal RGB filter (CRI).

### Statistical Analysis

Ultrasound echo signal increase of tumor regions after HerDox and Dox injection was evaluated for each group by the ultrasound echo signal of the tumor regions before drug injection as a reference *in vivo*. In addition, ultrasound echo signal of harvested tumors of mice receiving HerDox and Dox were compared to the signal of harvested tumors of mice without treatment *ex vivo*. All data are expressed as mean ± standard deviation of indicated sample sizes, and were analyzed by a two-sided paired t test, with the level of significance set at P = 0.05.

## Results

### High-frequency ultrasound imaging detects and monitors HerDox-mediated tumor cell death during treatment *in vivo*

Our previous studies on the therapeutic efficacy of HerDox entailed regular measurements of tumor growth during and after treatment over several weeks of tumor monitoring [26]. Here we examined the utility of ultrasound imaging for assessing whether immediate effects of HerDox treatment could be detected *in vivo* during treatment. Our previous study showed that 0.004 mg/kg HerDox is as effective as 10-fold higher [0.04 mg/kg] untargeted Dox on tumor ablation [26]. Therefore, these doses were chosen for the present study. Tumor-bearing mice received daily intravenous injections of HerDox (0.004 mg/kg/day) or Dox (0.04 mg/kg/day) for up to six days while ultrasound imaging of tumor regions was performed before drug administration, and after the third and sixth days of drug administration. Both the scattering area and intensity at tumor sites (indicated by arrows) increased with both HerDox and Dox treatment frequency [Fig. 2A and B, ultrasound images]. In contrast, the untreated tumors do not exhibit any significant increases (p = ∼0.95) (Fig. 2C). Quantification of scattering intensity (Fig. 2, graphs) showed that the average intensity of the tumor increased considerably after the third injection and increased nearly two-fold higher over untreated tumors by the sixth injection (HerDox: p = ∼0.0009, Dox: P = ∼0.0010). There were no significant differences in the average intensity values of between HerDox-treated and Dox-treated tumors after the sixth drug administration (p = 0.6097), suggesting that 0.004 mg/kg HerDox and 0.04 mg/kg Dox exhibit similar treatment efficacy on tumors.

**Figure 2:** High-frequency ultrasound imaging of tumor regions in mice receiving (A) 0.004 mg/kg/day HerDox or (B) 0.04 mg/kg/day Dox, by i.v. delivery and in (C) untreated mice: Ultrasound images of tumor regions were obtained after the indicated drug injection (before drug injection, after the third daily drug injection, and after the sixth daily drug injection) while mice received daily i.v. injections of the indicated drugs for six sequential days. Graphs (right-panel) depict average echo intensities of tumor regions (0, before drug injection; 3, immediately after the third daily drug injection; 6, 24 h after the sixth daily drug injection). *: p<0.01, +: p = ∼0.6097, and − : p = ∼0.95. The error bars indicate standard deviations. The arrows indicate tumor regions.

In order to verify the *in vivo* results, we performed high-frequency ultrasound imaging of tumors extracted from the same mice receiving daily HerDox and Dox injections for 6 days. The *ex vivo* imaging shows that the overall echo intensities of both HerDox [Fig. 3B] (p = 0.002) and Dox [Fig. 3C] -treated tumors (p = 0.003) are significantly higher than those of untreated -tumors [Fig. 3A]. Quantitatively, these intensities were nearly twice as high as those of the untreated tumors. Finally, as the source of this increase in echo intensity might be attributed to nuclear condensation and fragmentation in apoptotic cells [29]–[32], we examined the aforementioned tumors for apoptosis. After harvesting tumors from the same mice treated with HerDox and Dox for 6 days and the untreated mice, H&E stained and unstained sections of the tumors were prepared for histochemical assessment. The TUNEL images show that both HerDox and Dox treatments resulted in apoptotic marker elevation over tumors from un–treated mice (Fig. 4A). TUNEL fluorescence measurements of HerDox-treated tumors significantly differed (p<0.01) from those of untreated tumors (Fig. 4A, bar graph). In addition, greater nuclear shrinkage and fragmentation (arrows) could be observed in the H&E images of HerDox and Dox -treated tumors (Fig. 4B) than untreated tumors.

**Figure 3:** High-frequency ultrasound images of tumors *ex vivo* after extracting from mice treated with Dox and HerDox: Ultrasound images were obtained of tumors extracted from (A) an untreated mouse, (B) a mouse treated with 0.004 mg/kg/day HerDox, or (C) a mouse treated with 0.04 mg/kg/day Dox. (D) Echo signal intensities of A–C, respectively. The error bars reflect standard deviation. *: p<0.01.

**Figure 4:** TUNEL and H&E stained images of untreated, HerDox-treated, and Dox-treated tumors: (A) TUNEL images of untreated tumors (left), HerDox-treated tumors (middle) (injection drug dosage: 0.004 mg/kg×6 injections), Dox-treated tumors (right) (injection drug dosage: 0.04 mg/kg×6 injections) were acquired using confocal imaging (ex: 488 nm, em: 510–560 nm, and 10×) of tumor specimens. The arrows indicate the boundary between apoptotic and normal cells. Insets represent magnified images. (B) Average fluorescence of the TUNEL images of untreated, Dox-treated, HerDox-treated tumor sections (*: p<0.01) (C) H&E images of untreated (left), HerGa-treated tumors (middle), and Dox-treated tumors (right) were obtained using the Olympus microscope incorporating a CCD camera with a RGB filter (10×). The scale bar represents 200 µm. Arrows indicate nuclear shrinkage and fragmentation.

### Combining fluorescence intensity, *in situ* confocal, and spectral imaging modalities enables quantitative discrimination of HerDox fluorescence from autofluorescence

To assess whether HerDox could be detected in treated tumors at the cellular and subcellular level, and discriminate HerDox fluorescence from autofluorescence, we introduced high-resolution *in situ* confocal and ratiometric spectral imaging. The inherent fluorescence of Dox has the potential to enable studies in its biodistribution, depending on the dose of Dox and the sensitivity of the imaging system. In our previous studies, fluorescence intensity imaging allowed us to track the biodistribution of HerDox and demonstrate that HerDox undergoes tumor-specific targeting *in vivo*, in contrast to free, untargeted Dox [26]. In the present study, tumors and tissues extracted from mice 24 h after receiving daily i.v. injections of HerDox (0.004 mg/kg/day) for 6 consecutive days were examined by fluorescence intensity, *in situ* confocal, and ratiometric spectral imaging. The fluorescence intensities measured from tumors of HerDox-treated mice were over 50% higher than those measured from the liver, kidney, and skeletal muscle, while the heart and spleen exhibited no detectable fluorescence [Fig. 5A, left]. In situ confocal imaging [Fig. 5A, right] showed that the fluorescence intensity of tumor cells from HerDox-treated mice [Fig. 5A, right] was significantly higher than that of tumor cells from untreated mice [Fig. 5B]. Moreover, Dox fluorescence could be detected in the nuclei of HerDox-treated tumor cells, [Fig. 5A right, arrows], but not in the nuclei of untreated tumor cells [Fig. 5B]. In contrast, unlike in Fig. 5(A), we could not determine whether Dox fluorescence could be detected in the nuclei of Dox treated tumor cells. Here quantitative analysis (Fig. 5C) shows that the average fluorescence intensity of HerDox treated tumors is almost twice that of untreated tumors (p<0.01) as well as higher than that of Dox-treated tumors (p<0.01). Here, the standard deviation of fluorescence intensity for HerDox treated tumors is somewhat higher than others since there is considerable difference in fluorescence intensities between HerDox and non-HerDox regions, as shown in Fig. 5A and 5B. Thus, these results verify that the combination of these imaging modalities allows us to quantitatively assess tumor-accumulation of HerDox at cellular and sub-cellular levels in detail.

**Figure 5:** Fluorescence intensity image of harvested tissue *and in situ* confocal fluorescence of tumors: (A) Fluorescence image (left-panel; Ex: 532 nm; Em: 590±30 nm) of organs and tumors extracted from mice receiving HerDox (0.004 mg/kg/day; see Methods). Confocal fluorescence images of the tumors extracted from HerDox-treated (A, right-panel), Dox-treated (B, right), and untreated mice (B, left) were acquired at different z-depths (a total of thickness: 32 µm) with a step size of 2 µm. Maximum intensity z-projection of confocal fluorescence images of HerDox-treated and untreated tumors was performed. HerDox and Dox fluorescence in (A) and (B) are indicated by a color shift toward 255 on the scale bar in (A). The magnified image (A, right-panel) shows HerDox distribution in the tumor. Arrows indicate nuclei-localized fluorescence. (C) Mean fluorescence intensity of HerDox-treated, Dox-treated and untreated tumor. The error bar indicates standard deviation. *: p<0.01.

Ratiometric spectral imaging and analysis allowed discrimination between doxorubicin fluorescence of HerDox and autofluorescence in the same tumor areas. The reference spectral signatures [Fig. 6A, left] generated through the ratiometric method previously described (see Methods) show the relative HerDox contributions on the spectral signature of autofluorescence. The reference spectral signatures containing doxorubicin spectra with different ratios exhibit a peak at ∼590 nm, which is the typical maximum emission wavelength for HerDox, whereas the spectral signature of the autofluorescence exhibits no such peak at that wavelength [Fig. 6A, left]. The spectral classification images generated from these signatures [Fig. 6A, middle and right] clearly distinguished HerDox fluorescence from autofluorescence quantitatively and specifically, in spite of their strong spectral overlap. In particular, the classified image [Fig. 6A, middle] generated by four reference spectral signatures (cyan: 0.3·Dox+0.7·Autofl., red: 0.2·Dox+0.8·Autofl., blue: 0.1·Dox+0.9·Autofl., Green: Autofl.) allowed a greater degree of quantification than the classified image [Fig. 6A, right] generated by two reference spectral signatures (red: 0.2·Dox+0.8·Autofl. and Green: Autofl.) [25]. Moreover, the spectral unmixed image [Fig. 6B] shows HerDox localization in the tumor cells, in good agreement with the classified image by the two reference spectral signatures (red: 0.2·Dox+0.8·Autofl. and Green: Autofl.). Altogether, these findings show that spectral classification can discriminate doxorubicin fluorescence from autofluorescence, thus verifying that the tumor fluorescence detected here is indeed due to doxorubicin delivered by HerDox.

**Figure 6:** Ratiometric spectral classification images of HerDox-treated tumors *in situ:* (A) Ratiometric spectral classification images (middle and right-panel) of HerDox-treated tumors. Ratiometric spectral classification was performed using our previously developed program. Green: autofluorescence (Autofl.), Red: 0.2 Dox+0.8 autofl., Cyan: 0.3 Dox+0.7 autofl., and Blue: 0.1 Dox+0.9 autofl.. The reference spectral signatures used to generate the spectrally classified image are shown in the left-panel. (B) Spectral unmixed image. Scale bar: 80 µm.

## Discussion

We designed this study to take advantage of the specific strengths of several complementary non-invasive imaging methods, used in a concerted (multimodal) way, in order to achieve better quantification and understanding of targeted therapy-relevant events in living animals, with ultimately translational purposes. The imaging modalities utilized in this study have provided multiple and complementary information in the assessment and characterization of our nanoparticles. Through these studies, we have observed that 1) high frequency ultrasound imaging allows us to quantitatively assess nanoparticle efficacy at micro scales, particularly tumor cell apoptosis, by resolving micro-anatomy of tumor regions non-invasively. In contrast, standard optical imaging technologies typically require contrast agents in order to investigate tumor cell apoptosis *in vivo* [33]; 2) fluorescence intensity and confocal imaging enables us to verify the tumor targeting capacity of the nanoparticles at macro-to-micro scales; 3) ratiometric spectral imaging allows us to discriminate between Dox fluorescence and autofluorescence more quantitatively and specifically, thus verifying the results obtained by using the fluorescence intensity and confocal imaging *ex vivo*. In particular, the methods, including confocal imaging and ratiometric spectral imaging, complement one other: while confocal fluorescence imaging provides insight into the local densities of Dox distributions over cells by fluorescence difference in detail, ratiometric spectral imaging, which typically is less sensitive to local densities of fluorescent molecules, offers quantitative discrimination between autofluorescence and Dox fluorescence. In addition, confocal imaging offers more details than standard fluorescence imaging of small animals or tissues, thus enabling monitoring of Dox distributions over tumor cells at sub-micron scales. Taken together, these imagaing modalities complement one another when used in combination and provide multiple types of information in the characterization of the nanoparticles during preclinial asessement.

Previous studies have reported that cell death could be monitored using high-frequency ultrasound imaging [29]–[32]. Those studies showed that the ultrasound echo intensity of tissues was increased by cell apoptosis *in vivo* and *ex vivo*, and attributed this increase in echo intensity to nuclear condensation and fragmentation in apoptotic cells [29]–[32]. In the present study, we could observe that the average intensity of the tumor increased considerably after the third injection and increased significantly over untreated tumors by the sixth injection of HerDox. In these experiments, the ultrasound images obtained before HerDox and Dox injection were utilized as negative controls. In addition, the *in vivo* and *in vitro* results in Fig. 2C and 3 show that the untreated tumors still exhibit lower echo signals than the HerDox and Dox-treated tumors, thus indicating that the ultrasound echo signal changes of untreated tumors within 6 days can be negligible compared to the changes by HerDox and Dox treatment. In agreement with these findings, the same tumor tissue yielded a positive TUNEL signal, showing that apoptosis was induced by drug treatment. The significant differences between the volumes of drug-treated and untreated-tumors, which were measured using calipers, were ascertained after monitoring tumor growth for up to 25 days following the drug administration in our previous studies [26]. In contrast, high-frequency ultrasound imaging used here enabled us to distinguish the echo intensity increase in the tumor regions *during* tumor treatment, thus assessing the trajectory of therapeutic efficacy much earlier. It is important to note that HerDox and Dox are incapable of inherently causing any significant increase of ultrasound echo signal because their sizes (less than 40 nm) are significantly smaller than the ultrasound wavelength.

Our previous studies have assessed the tumor targeting capacity of HerDox *in vivo* by using fluorescence intensity imaging [26], which has allowed us to understand how HerDox reaches tumors and accumulates in them. In those studies, the dose required for monitoring biodistribution of HerDox was nearly five-times the therapeutic dose, as the therapeutic dose falls below the level of detection for biodistribution and pharmacokinetic studies because of the inherent weak fluorescence of Dox [26]. The multimodality imaging system utilized here offers highly-sensitive fluorescence intensity imaging, thus allowing us to detect sub-nano molar cocentrations of Dox *in vitro*. Using the multimodality imaging in the present study, we could observe tumor accumulation of HerDox after multiple delivery at therapeutic doses *in vivo*. Moreover, cellular accumulation could be observed and quantitatively measured at the cellular and subcellular level using confocal imaging (detection limitation: ∼0.1 nM). In our prevous *in vitro* stuides, we could observe that doxorubicin is localized in the nucleus of HerDox and Dox-treated cells [26]. Here we could also observe that Dox fluorescence could be found in the nuclei of HerDox-treated cells. However, unlike HerDox-treated tumor cells [Fig. 5(A)], we could not easily determine whether Dox is localized in nuclei of the Dox treated tumor cells since the nuclei localization could not be easily determined, likely due to cytoplasm collapse [Fig. 5(B)]. While nuclear counter-staining, such as DAPI, can be used to verify the localization of Dox in the tumor cells, this was not performed because in situ confocal imaging of fresh, non-processed, unstained tumors took place immediately after tumor extraction. In general, non-viable cells exihibit stronger autofluorescence than viable cells [34]. In the present study, we could observe that the fluorescence emitted from HerDox-treated tumors was nearly two-fold over the autofluorescence from untreated tumors (Fig. 5C). The TUNEL assay [Fig. 4.(a)] verified tumor cell apoptosis following HerDox treatment. In addition. ratiometric spectral classification and spectral unmixing allowed us to distinguish emissions due to HerDox fluorescence and autofluorescence (Fig. 6). Based on these distinctions, our data suggest that the increased fluorescence from the HerDox-treated tumor is likely to result from both HerDox accumulation and cell death rather than just the increased autofluorescence caused by cell death alone. Hence, the combination of confocal and spectral imaging allows discrimination between Dox fluorescence and autofluorescence quantitatively. Taken together, our approch shown here may also provide a better understanding of how HerDox reaches tumors and achieves deposition of the drug payload to the tumors.

In conclusion, the multimodal imaging approach used here, which includes high-frequency ultrasound, fluorescence intensity, confocal, and spectral imaging, has allowed us to assess the efficacy of our novel tumor-targeted chemotherapeutic nanoparticle, HerDox, thus providing an alternative method to the established assessments of targeted therapeutic efficacy. The combination of imaging modalities enables monitoring of tumor cell death *during* HerDox treatment *in vivo*, in contrast to standard measurements of tumor growth over time that delay such assessment until some time after treatment. Overall, this may greatly shorten the time required for assessing preclinical efficacy. Also, it enables discerning and documenting of HerDox localization in tumors *in situ* with high resolution, quantitatively and specifically. One may envisage using this approach to screen a panel of new nanotherapeutics *in vivo* in order to select one for more expanded testing of therapeutic efficacy. Such an approach may enhance the efficiency and accuracy of preclinical evaluation of new nano-molecules, thus reducing time and cost for the translation of new nanotherapeutics into the clinic as well as providing better cancer treatments. Since the techniques described here, including fluorescence intensity, confocal, and spectral imaging, are aimed at fluorescence-based assessments, most therapeutic molecules would require labeling with a fluorophore. This is not unusual, and in fact, many researchers characterizing nanotherapeutic particles *in vivo* have attached fluorophores to their particles to visualize localization *in vivo*. Whether the molecules of interest are inherently fluorescent, such as the HerDox molecule described here, or labeled with a fluorophore, the multimodality imaging method described here can provide a powerful approach for characterizing nanoparticle activities *in vivo* in preclinical studies.
